RETRACTED

# TET1 exerts its tumour suppressor function by regulating autophagy in glioma cells

**DOI:** 10.1042/BSR20160523

**Published:** 2017-11-06

**Authors:** Rui Fu, Yan Ding, Jie Luo, Li Yu, Cheng Lin Li, Dong Sheng Li, Shi Wen Guo

**Affiliations:** 1 Department of neurosurgery, affiliated Taihe hospital of Xi’an Jiaotong University Health Science Center, Shiyan, Hubei, China; 2 Hubei Key Laboratory of Embryonic Stem Cell Research, Taihe Hospital, Hubei University of Medicine, Shiyan, Hubei 442000, China

**Keywords:** autophagy, CRISPR/Caspase-9, glioma, methylation, TET1

## Abstract

DNA methylation and demethylation play a critical role in the regulation of the molecular pathogenesis of gliomas. Tet methylcytosine dioxygenase 1 (TET1) catalyses the sequential oxidation of 5-methylcytosine (5mC) to 5-hydroxymethylcytosine, (5hmC) leading to eventual DNA demethylation. It has been reported that TET1 is a tumour suppressor in several cancers. However, whether TET1 plays a role in glioma development is largely unclear. Different glioma specimens and corresponding normal controls were collected to analyse the expression of TET1. At the same time, TET1 of glioma U251 cells was knocked down or overexpressed to observe its effect on glioma cell proliferation and invasion as well as autophagy level. Here, we reported that the expression of TET1 in glioma tissue was significantly lower than the corresponding non-tumour normal tissues, and the concentration of TET1 is negatively correlated with the glioma WHO classification. When *TET1* gene in glioma U251 cells was knocked down by CRISPR/Caspase-9 system, the proliferation and invasive ability of U251 increased remarkably. But when TET1 was overexpressed in U251 cells, the proliferation and invasion were impaired. Following the down-expression of TET1, the level of autophagy in U251 cells decreased accordingly.However, when TET1 was overexpressed in U251 cells, the level of autophagy incraesed. Furthermore, bafilomycin A1 (Baf-A1) but not 3-methyladenine (3-MA) could decrease the autophagy level of TET1^−/−^ U251 cells as the wild-type controls. It suggests that the tumour suppressor effect of TET1 seems to be mediated by regulating the level of autophagy, and the regulation of TET1 on autophagy is at an early stage.

## Introduction

Glioblastoma (GBM) is one of the most common and malignant tumours of the central nervous system, characterized by adaptation to poorly immunogenic and hypoxic conditions. Despite advances and progress in surgery, chemotherapy and radiation, the average survival time of patients suffering from GBM is only 9–12 months and the progression-free survival (PFS) time is approximately 5–8 months [1–3]. Increasing evidence suggests that the major obstacle to effective treatment of gliomas is the highly proliferative, migrative and invasive nature of glioma cells [4]. However, the mechanisms underlying these cellular events are still poorly understood. Therefore, understanding the regulatory mechanisms involved in these biological characteristics of GBM cells is essential for developing novel and effective therapeutic approaches.

RETRACTED

DNA methylation and demethylation play crucial roles in many biological processes, including regulation of gene expression, maintenance of genomic stability and integrity. Studies in cancer biology revealed that DNA methylation plays a determinant role in silencing of oncogenes during cancer development, suggesting that DNA methylation and demethylation may play important roles in various physiological processes other than housekeeping-like functions such as maintaining genome stability [5].

Previous studies showed that the Tet methylcytosine dioxygenase 1 (TET1) protein could catalyse the conversion of 5-methylcytosine (5mC) of DNA to 5-hydroxymethylcytosine (5hmC), resulting in DNA demethylation [6]. However, whether TET family proteins may be involved in the tumorigenesis of glioma cells is not clear.

## Materials and methods

### Cell culture

Human glioma U251 cells were preserved in our laboratory,and were maintained in Dulbecco’s modified Eagle medium (DMEM, Gibco, U.S.A.), supplemented with 10% FBS (Invitrogen, Carlsbad, CA, U.S.A.) and 1% P/S solution (100 units/ml penicillin, 100 mg/ml streptomycin). Cells were habitually passaged at 3–4 day intervals in a humidified atmosphere of 5% CO_2_ at 37°C.

### Immunohistochemistry

Different glioma specimens (ten for each grade) were collected from patients who underwent resection of gliomas between 2013 and 2015 at Taihe Hospital, The Affiliated Hospital of Hubei University of Medicine. The histological type of gliomas was determined according to WHO classification criteria and the immunohistochemistry was performed as described in our previous study [7].

### CRISPR vector and single-guide RNA cloning

The pGK1.2 vector (Genloci, China) expressing Caspase-9 and containing a cloning site for the single-guide RNA (sgRNA) sequence was digested with BbsI (NEB). TET1 sgRNAs were constructed online (http://crispr.mit.edu/) and then cloned into the pGK1.2 vector according to the manufacturer’s instructions. The complementary oligos with two overhanging sequences CACC or AAAC at 5′ for each sgRNA were annealed to form double-stranded sequence and finally ligated with the linearized pGK1.2. Competent cells were transformed with 2 μl of the ligated plasmid and plated in LB plates with selection. The single colonies were expanded prior to plasmid extraction using Maxiprep kit (Qiagen). The correct insertion of the sgRNA sequences was confirmed using Sanger sequencing.

RETRACTED

### TET1 overexpression

Plasmid construction of TET1 overexpression plasmid was constructed with pCAG-transcription activator like effector (TALE)-VP63-IRES-PuroR, which contains a TALE system and an VP64 activator. TALE is responsible for recognizing the target sequence and VP64 is used to activate the expression of TET1. The selection of the target sequence and the construction of the plasmid were performed according to the manufacturer’s instructions.

### Selection of TET1 mutation corrected U251 clones

U251 cells were transfected using the Amaxa cell line Nucleofector Kit V (Lonza) according to manufacturer’s guidelines, and 1 × 10^6^ cells were transfected with 10 μg of pGK1.2 plasmid and then transfected for the second time after 24 h. Puromycin (3 μg/ml) was used to select the positive cells. After 3 days of selection, cells were plated in 96-well plates and incubated at 37°C for 2 weeks before harvesting for DNA extraction. The percentage of TET1 targeting were analysed with T7 endonuclease 1 (T7E1) as described in our previous study [7].

### Cell growth assay

The proliferation capability of U251 cells were detected with RTCA DP Analyzer (ACEA). U251 cells with or without TET1 disruption were digested with 0.05% trypsin-EDTA and plated into E-Plate 16 at a density of 1 × 10^3^/well and incubated at 37°C for 140 h. The experiment was performed in triplicate.

### Invasion assay

The invasion ability of U251 cells was analysed with Transwell filters as described in our previous study [7]. The upper surface of Transwell filter (Millipore, Billerica, MA, U.S.A., diameter: 12 mm, pore size: 8 mm) was coated with Matrigel, and then 1 × 10^5^ cells suspended in serum-free medium were plated into the top side of the polycarbonate. Medium with serum was used as a chemoattractant in the lower chamber. The cells were incubated at 37°C for 48 h before removing the medium from the top chamber. The non-migratory or non-invasive cells were scraped off with a cotton swab. Cells on the lower surface were fixed in 70% ethanol for at least 10 min, then washed and stained with 0.1% Crystal Violet for 5–10 min. Images were collected under an inverted microscope (Olympus) and the number of migrated cells were counted. Each assay was repeated three times.

### Chemical treatments of U251 cells

U251 cells were stabilized in corresponding medium. For induction of autophagy, U251 cells were cultured in EBSS buffer for 24 h. For inhibition of auotphagy, U251 cells were cultured in medium supplemented with 10 mM 3-methyladenine (3-MA) or 2 μM bafilomycin A1 (Baf-A1) for 24 h.

RETRACTED

### Autophagosome detection

U251 cells were fixed with 4% paraformaldehyde for 30 min, then washed and stained with 0.1% Acridine Orange for 5–10 min. Images were collected under a fluorescence microscope (Leica).

### Western blot

Proteins from cells (40 μg/lane) were separated by SDS/PAGE (10% gel) before transferring on to a nitrocellulose (NC) membrane (Millipore). Membranes were blocked by 5% skim milk at room temperature for 1 h, and then incubated overnight at 4°C with primary antibody. The primary antibodies and dilutions used were as follows: GAPDH (Beyotime, AG019, 1:500), LC3B (Beyotime, AL221, 1:1000), mTOR (Beyotime, AM832, 1:1000), Beclin 1 (Cell Signaling Technology, 3495S, 1:200, Danvers, MA, U.S.A.) and TET1 (Santa Cruz, sc-163443, 1:200). After rinsing for three times using slow shaking for 5 min each time with TBST, the membranes were incubated with alkaline phosphatase–conjugated goat anti-rabbit or anti-mouse IgG (Beyotime, 1:1000, China) for 2 h at room temperature followed by three times washing with TBST. At last, the membrane was visualized with the BCIP/NBT Alkaline Phosphatase Color Development Kit (Bio–Rad ChemiDoc XRS, U.S.A.). GAPDH was used as the loading control in the Western blots.

### Statistical analysis

All data were expressed as mean ± S.D. Statistical analyses were performed with the Student’s *t* test by using GraphPad Prism 5. Statistical significance will be considered when *P-*value is <0.05.

## Results

TET1 expression correlated with malignancy and prognosis in glioma patients. TET1 expression in glioma specimens and adjacent non-cancer tissues from 30 patients with glioma (ten for each grade specimen) was detected by immunohistochemistry. The expression of TET1 was highly expressed in adjacent normal tissue and could be detected in almost 80% of WHO grade II and 50% grade III glioma specimens. On the contrary, TET1 could hardly be detected in WHO grade IV glioma specimens (Figure 1A,B). We also detected the expression of TET1 in glioma cells U251, DBTRG and U87-MG. It was shown that the expression levels of TET1 in glioma tissue were also significantly lower than that of normal human glial cells. This indicated that the expression of TET1 was negatively correlated with clinical grading and malignant degree of glioma (Figure 1C,D).

**Figure 1:** TET1 expression correlated with malignancy of glioma. The expression levels of TET1 in glioma specimens and glioma cell lines. (**A**) Immunohistochemistry detection of the expression of TET1 in different grades of glioma tissues (ten for WHO II–IV and adjacent tissues respectively). The left panel showed adjacent tissues and the right panel presented glioma tissues. (**B**) Histogram showed the percentage of TET1-positive specimens; (**C**) RT-PCR detected the expression of TET1 in different glioma cell lines; (**D**) Western blot detected the expression of TET1 in different glioma cell line U251, DBTRG and U87-MG; ^#^*P*<0.05.

RETRACTED

### TET1 CRISPR/Caspase-9 plasmid construction and transfection

To investigate the role of TET1 in glioma cells, CRISPR/Caspase-9 technology was applied to knockout TET1 of glioma cells. TET1 sgRNAs were designed on http://crispr.mit.edu/, 3 score >95 sgRNAs were selected to construct TET1 CRISPR/Caspase-9 plasmid. Through activity detection, sgRNA#3 was the highest and selected for the following study (Figure 2A). TET1 CRISPR/Caspase-9 plasmid was transfected into U251 cells with an electrical transfection instrument NEPA21 (Japan) as previously described (Figure 2B) [7]. T7E1 was used to analyse the targeting efficiency of TET1 CRISPR/Caspase-9, and it was found that the targeting efficiency was more than 30% (Figure 2C). Single cell culture was used to select the TET-knockout colons. Screened by sequencing, one clone with biallelic TET1 mutations was selected and used for the next study (Figure 2D).

**Figure 2:** TET1 CRISPR/Cas9 plasmid construction and the effects of TET1 knockdown on U251 cells. CRISPR/Cas9 mediated *TET1* gene targeting in U251 cells and the effects of TET1 knockdown on U251 cells. (**A**) Diagrammatic sketch of TET1 and its target site by CRISPR/Cas9 plasmids. (**B**) Fluorescence microscopic observation of the transfection efficiency of CRISPR/Cas9 plasmids. Cells with green fluorescence were positively transfected ones. (**C**) CRISPR/Cas9 targeting detection. After two rounds of targeting by CRISPR/Cas9, the target sites of TET1 were amplified by PCR and then digested by T7E1 to evaluate the proportion of the mutated TET1. (**D**) Sequencing of TET1 for the selected cell clone after two rounds of targeting by CRISPR/Cas9. (**E**) xCELLigence RTCA detection was used to test the cell viability. Green one is the TET1^−/−^ group and the red one represents the wild-type group (*P*<0.05). (**F**,**G**) Transwell tests the invasion ability of TET1^−/−^ and wild-type cells. The Crystal Violet staining positive cells were those that passed through the Matrigel and Transwell (F). These cells were counted under an inverted microscope, and the numbers were shown in the histogram (G). (**H**) Western blot detected the level of autophagy in different groups. LC3B, Beclin 1 and P62 were detected. (**I**,**J**) Acridine Orange staining detected the autophagosomes in TET1^−/−^ and wild-type U251 cells. The orange fluorescence presents the autophagosomes (I); and the numbers of autophagosomes were shown in the histogram (J); *P<0.05.

RETRACTED

Knockdown of TET1 facilitates cell viability and invasion of U251 cells. xCELLigence RTCA DP Instrument (ACEA Biosciences, RTCA DP, U.S.A.) was used to test the viability of cells. TET1 targeted and wild type U251 cells were plated into an E-Plate 16 plate respectively, at a density of 1 × 10^3^/well and monitored for 120 h. Each group was performed in triplicate. The results of the cell viability increased in the TET1-disrupted group as compared with the control from 2 to 5 days (Figure 2E, *P*<0.05). These results indicated that down-regulation of TET1 could increase the viability of glioma cells.

To test whether TET1 indeed participates in the invasion, we performed Transwell assay with Matrigel to detect the invasion ability. As shown in Figure 2F,G, the TET1^−/−^ markedly increased the invasion rates of glioma cells as shown in the photography and quantificative analysis. In U251 cells, the number of cells that pass through the transwelll in the TET1^−/−^ cells and wild-type cells were 216 ± 23 and 138 ± 15 (*P*<0.05) respectively. This suggested that the down-regulation of TET1 could facilitate the migration ability and invasion ability of glioma cells.

TET1 regulates autophagy in U251 cells. To determine the possible mechanisms of TET1 in regulating glioma cell malignancy behaviour, we detected the expression level of pluripotency-associated proteins, autophagy factors and apoptosis proteins. It was found that the autophagy level was decreased in TET1^−/−^ U251 cells. Western blot showed that LC3B and Beclin 1 levels were decreased, while P62 was increased in TET1^−/−^ group compared with wild-type controls (Figure 2H). Moreover, Acridine Orange staining indicated that the number of autophagosomes in the TET1^−/−^ group was also lower than that of control (Figure 2I,J).

To further test the regulation of TET1 on autophagy, EBSS, 3-MA and Baf-A1 were used to induce or inhibit autophagy. It was found that the sensitivity of U251 cells to EBSS was affected by TET1 expression (Figure 3A) and Baf-A1 but not 3-MA that could decrease the autophagy level of TET1^−/−^ U251 cells as the wild-type controls (Figure 3B).

**Figure 3:** The effect of TET1 expression on the autophagy of U251 cells . The effect of TET1 expression on the sensitivity of U251 cells to autophagic inducer and inhibitors. (**A**) After treating with EBSS for 6 h, Western blot detected the level of autophagy in different groups. (**B**) After treating with 3-MA (10 mM) or Baf-A1 (2 μM) for 24 h, Western blot detected the level of autophagy in different groups. LC3B and Beclin 1 were detected.

RETRACTED

TET1 overexpression impeded cell viability and invasion and increased autophagy of U251 cells. Six target sequences before the TET1 transcriptional start site were selected (Supplementary Figure S1A). After plasmid construction, the identification activity showed that all the six plasmids could increase the expression of TET1 by 2-5 times, and plasmid WX1402-2 had the highest activity (Supplementary Figure S1B), which was selected for the subsequent study.

Plasmid WX1402-2 was transfected into the U251 cells by Lipofectamine® 3000 Transfection Reagent (Invitrogen, LP3000-015). Puromycin was used to select the positively transfected cells. After 10 days of selection culture, five single cell clones were screened. RT-PCR and Western blot were used to test the overexpression of TET1. It was found that two of them (clone 1 and clone 2) were TET1-overexpressed, and both of them were in the following studies (Supplementary Figure S1C).

Cell activity analysis showed that the activity of both clone 1 and clone 2 was lower than the wild group (Figure 4A). Transwell assay indicated that compared with the wild-type controls (145 ± 18), the number of cells that invaded the Matrigel and passed through the transwell micropore in the clone 1 and clone 2 were both decreased, which were 86 ± 10 and 91 ± 11 respectively (Figure 4B,C).

**Figure 4:** The effect of TET1 overexpression on the viability and invasion of U251 cells. TET1 overexpression impeded cell viability and invasion of U251 cells. (**A**) xCELLigence RTCA detection showing the cell viability of clone 1, clone 2 and wild-type cells from 0 to 140 h. Green one is wild-type group, red and blue represent clone 1 and clone 2 respectively (*P*<0.05). (**B**,**C**) Transwell detection of the invasion ability of clone 1, clone 2 and wild-type cells. The Crystal Violet staining positive cells were those that passed through the Matrigel and Transwell (B). The Crystal Violet staining positive cells were counted under the inverted microscope, and the numbers were shown in the histogram (C).

To further verify the relationship between TET1 and autophagy, we detected the autophagy level of clone 1 and clone 2. Consistent with the previous study, Western blot showed that the level of LC3B and Beclin 1 were decreased in clone 1 and clone 2 (Figure 5A), and the number of autophagosomes in both of them was also lower than that of control (Figure 5B,C). The same phenomenon was observed in another glioma cell line DBTRG (Supplementary Figure S2).

**Figure 5:** The effect of TET1 overexpression on the autophay level of U251 cells. TET1 overexpression correlated with autophagy in U251 cells. (**A**) Western blot detection of the autophagy levels in different groups. LC3B, Beclin 1 and P62 were detected. (**B**,**C**) Acridine Orange staining detection of the autophagosomes in clone 1, clone 2 and wild-type U251 cells. The orange fluorescence presents the autophagosomes (B); and the numbers of autophagosomes were shown in the histogram (C); ^#^*P*<0.05.

RETRACTED

## Discussion

TET1 is one of the human TET family proteins, which catalyses the conversion of 5mC into 5hmC [6]. Recently, the role of TET proteins in 5hmC correlated to diseases has been widely studied. It was suggested that TET1 was lost or less expressed in diverse solid tumours including human colon, gastric, liver cancers and breast tumour [8–11]. Furthermore, previous studies demonstrated that the 5hmC levels were reduced in a small series of astrocytomas and GBMs as compared with normal brain [12–14]. However, whether TET1 is associated with the malignance of glioma and the mechanism underlying them are not clear.

In the present study, we investigated expression levels and biological function of TET1 in human glioma tissue and U251 cells. It was shown that the expression level of TET1 was lower in cancre cells than in the normal control. TET1 CRISPR/Caspase-9 and TALE-VP64 plasmids were used to mediate the knockdown and overexpression of TET1, and then for further determination of biological function. It was found that cells with TET1 knockdown showed lower levels of 5hmC, which might contribute to aberrant DNA methylation patterns or other aspects in cancers. Moreover, the TET1 knockdown resulted in the growth stimulation and increased invasion, while the TET1 overexpression resulted in reverse. These data indicated that TET1 is an important regulator and TET1 mutations or dysregulation might lead to lethality.

Autophagy is a biological process that mediates degradation of large number of small proteins and old or damaged organelles [15,16]. It is also linked to cell death and is known as type II programmed cell death mechanism [17]. The exact mechanism of autophagic cell death is not known and is an interesting topic for investigation. Autophagy has been shown to promote or inhibit tumorigenesis based on the tumour type and stage [18,19]. The role of autophagy in glioma genesis is not well understood. In the present study, to investigate mechanism of TET1-mediated tumour suppressor, we tested the expression levels of autophagy genes in TET1 up- and down-regulated U251 cells. It was found that the expression level of Beclin 1 and LC3B were lower in TET1 knockdown group but higher in TET1 overexpression group than that of the wild group. Acridine Orange staining showed that the number of autophagosomes were lower in TET1 knockdown group but higher in TET1 overexpression group than the wild group. It suggested that the autophagy level was negatively related to TET1. Furthermore, when treated with EBSS, 3-MA or Baf-A1, the autophagy was more sensitive in TET1^−/−^ U251 cells when compared with wild-type cells and Baf-A1 but not 3-MA could decrease the autophagy level of TET1^−/−^ U251 cells as the wild-type controls. It suggested that the regulation of TET1 on autophagy is at an early stage.

RETRACTED

Cell migration and invasion are highly regulated processes involved in physiological and pathological conditions. Reports have shown that the higher expression levels of the pivotal autophagy genes, *LC3* and *Beclin1*, correlate with the better survival of GBM patients [20], suggesting the growth inhibitory effect of autophagy in GBM. Furthermore, a growing number of studies show that methylation existed in many tumour autophagy regulatory genes, such as *mTOR* [21] and *Beclin1* [22], suggesting that the autophagic process is required for glioma cells to migrate, and the down-regulation of some autophagy genes limits migration and invasion capabilities of glioma cells [23,24]. However, it is also reported that during autophagy occurrence, (GBM) migration and chemokine-mediated invasion were both impaired, but in Beclin 1-silenced GBM cells, an increased migration capability was observed [25]. From what has been discussed above, we speculated that the tumour suppressor role of TET1 was mediated by regulating autophagy.

## Conclusion

Our data suggested that TET1 plays an important role in the development of GBM by regulating the level of autophagy.

## Availability of data and materials section

The datasets and/or analysis of the present study are available from the corresponding author on reasonable request.

## Supporting information

## Abbreviations

Baf-A1: bafilomycin A1
CRISPR: Clustered regularly interspaced short palindromic repeats
EBSS: Earle’s Balanced Salt Solution
GAPDH: glyceraldehyde-2-phosphate dehydrogenase
RT-PCR: Reverse transcription- PCR
mTOR: mammalian target of rapamycin
GBM: glioblastoma
sgRNA: single guide RNA
TALE: transcription activator like effector
TET1: Tet methylcytosine dioxygenase 1
T7E1: T7 endonuclease 1
3-MA: 3-methyladenine
5mC: 5-methylcytosine
5hmC: 5-hydroxymethylcytosine
